# LncRNA ABHD11-AS1 Participates in the Progression of Cervical Carcinoma by Targeting miR-1254 and Is the Key to the Diagnosis and Treatment of Cervical Carcinoma in the Future

**DOI:** 10.1155/2022/8387458

**Published:** 2022-02-10

**Authors:** Duanrong Zhu, Qun Hao, Min Qian, Yuli Hu, Feifei Wu

**Affiliations:** Department of Obstetrics and Gynecology, General Hospital of the Eastern Theater Command, Nanjing 210002, Jiangsu, China

## Abstract

Cervical carcinoma is the most common gynecologic tumor in the clinic. The incidence of cervical carcinoma has been increasing in recent years, and the age of the affected population is showing a younger trend. Long-chain noncoding RNA (LncRNA) acts in the cell cycle. In cervical carcinoma, many studies have also confirmed the important role of LncRNA. LncRNA ABHD11-AS1 is one of the genes abnormally expressed in cervical carcinoma, but the specific situation has not been fully explained. This study intended to confirm whether LncRNA ABHD11-AS1 can be applied for the treatment of cervical carcinoma in the future. From January 2015 to January 2017, 72 cases of cervical carcinoma patients and 78 cases of healthy people during the same period in our hospital were selected for prospective analysis. ABHD11-AS1 and miR-1254 in serum and carcinoma tissues of cervical carcinoma patients were detected. In addition, human cervical carcinoma cells HeLa and CaSki were obtained to analyze the effects of interference with ABHD11-AS1 and miR-1254 on the biological behavior of cervical carcinoma cells. Finally, the correlation of ABHD11-AS1 with miR-1254 was verified by double fluorescein reporter enzyme and immunocoprecipitation. ABHD11-AS1 was upregulated, and miR-1254 was reduced in serum and carcinoma tissues of cervical carcinoma patients (*P* < 0.05). The expression levels of the two were negatively correlated (*P* < 0.001). ABHD11-AS1 decreased and miR-1254 increased in serum of cervical carcinoma patients after treatment (*P* < 0.05). High ABHD11-AS1 and low miR-1254 had a close correlation with the poor prognosis of cervical carcinoma patients (*P* < 0.05). Silencing LncRNA ABHD11-AS1 could inhibit the activity of cervical carcinoma cells (*P* < 0.05), while inhibiting miR-1254 could promote the activity of cervical carcinoma cells (*P* < 0.05). ENCORI online website found that LncRNA ABHD11-AS1 and miR-1254 had binding sites. Bifluorescein reporter enzyme experiment found that ABHD11-AS1-WT fluorescence activity was inhibited by transfected miR-1254-mimics (*P* < 0.05). LncRNA ABHD11-AS1 accelerates proliferation, invasion, and migration of cervical carcinoma cells through targeted regulation of miR-1254, which may become the key to the treatment of cervical carcinoma.

## 1. Introduction

Cervical carcinoma has had a rising incidence rate in recent years, and the age of the affected population is showing a younger trend [1, 2]. Cervical carcinoma is the biggest killer of women life and health. A survey shows that more than 200,000 people die from cervical carcinoma every year [3]. Therefore, an in-depth understanding of the pathogenesis of cervical carcinoma is helpful for the treatment of cervical carcinoma.

Through long-term efforts in clinical medicine, we have learned that the occurrence and progression of cervical carcinoma have a close correlation with proliferation, invasion, and migration of carcinoma cells [4]. However, it is still unclear what exactly affects the activation of carcinoma cells. In recent years, researchers at home and abroad have agreed that LncRNA acts in the cell cycle [5, 6]. However, in cervical carcinoma, many studies have also confirmed the important role of LncRNA [7, 8]. Recently, we found that LncRNA ABHD11-AS1 was involved in the occurrence and progression of endometrial carcinoma and also has a regulatory effect on the biological behavior of endometrial carcinoma cells [9]. Its clinical significance mainly lies in the fact that the early screening of tumor diseases still relies mainly on the traditional carcinoma markers CEA and CA199, which cannot accurately respond to complex tumor types, and more and more research studies also show that they can cause abnormalities of carcinoma markers. Later, we further consulted relevant studies. Liu et al. [10] found LncRNA ABHD11-AS1 was one of the genes abnormally expressed in cervical carcinoma during gene screening, but the specific situation has not been fully explained. Therefore, in order to confirm the situation of LncRNA ABHD11-AS1 in cervical carcinoma and its related mechanism, we first analyzed the downstream genes with binding sites with LncRNA ABHD11-AS1 through ENCORI and found that they include miR-1254. However, miR-1254 has been found to participate in cervical carcinoma by Zhou et al. [11]. LncRNA regulates the activities of cells through various ways and methods such as transcription in upstream promoter region, inhibition of RNA polymerization, and combination. At present, LncRNA has been proved to have participated in many tumor disease cells such as colon carcinoma, gastric carcinoma, and lung carcinoma [12–14]. Therefore, we preliminarily speculated that LncRNA ABHD11-AS1 may affect the process of cervical carcinoma through miR-1254. In order to verify our conjecture, we will carry out an experimental analysis to confirm whether LncRNA ABHD11-AS1 can be applied for the treatment of cervical carcinoma in the future.

## 2. Experimental Preparation

### 2.1. Research Participants

#### 2.1.1. Patient Data

From January 2015 to January 2017, cervical carcinoma patients and healthy people during the same period in our hospital were selected for prospective analysis. There were 72 cervical carcinoma patients (patients were 30–70 years old; patients were diagnosed as cervical carcinoma; patients were confirmed as early stage according to AJCC TNM staging standard; after admission, patients received neoadjuvant chemotherapy and radical tumor resection; patients or their immediate family members have signed informed consent forms; patients complicated with other severe diseases; patients have received radiotherapy, chemotherapy, surgery, and antibiotic treatment within half a year before admission; patients with autoimmune defects, with organ dysfunction, with low compliance, and with drug allergy were excluded; patients transferred from the other hospital were excluded) and 78 healthy people (patients aged 30–70 years; no major medical history was found; patients were informed and agreed to participate in this investigation). There was no statistical difference in baseline data such as age and sex between the two groups (*P* < 0.05). This experiment was carried out according to the Declaration of Helsinki. All patients signed informed consent forms, and the study was approved by the ethics committee.

### 2.2. Cell Data

HeLa, CaSki, and HcerEpic were obtained from ATCC. They were cultured in 90% DMEM high sugar medium containing glutamine and sodium pyruvate and 10% FBS and stored at 37°C with CO_2_.

## 3. Experimental Methods

### 3.1. Human Sample Collection

A 3 ml of fasting venous peripheral blood was obtained from cervical carcinoma patients at admission, at discharge, and during physical examination of healthy people, respectively, and serum was obtained by centrifugation. In addition, with the consent of the patient, the tumor tissue and adjacent tissue (more than 5 cm away from the carcinoma tissue) of cervical carcinoma patients during biopsy were obtained for subsequent detection. The patients were followed up for 3 years after discharge. The follow-up was carried out by hospital reexamination. The survival of the patients in this study was recorded, and the survival curve was visualized.

### 3.2. Cell Passage

The original culture solution was absorbed. The cells were rinsed twice with PBS, added with 6 mL (100 mm each dish) pancreatin, and observed under the microscope. When cells have just fallen off, the pancreatin was absorbed and left for about 0.5 mL, moved to the incubator for digestion, and taken out after 3 min. Passage was carried out using 12 mL of CM1-1 culture solution (90% DMEM high sugar culture solution containing glutamine and sodium pyruvate +10%FBS) to terminate digestion. The cells were gently blown evenly, and then divided into 3–6 dishes for culture.

### 3.3. Cell Transfection

Cervical carcinoma cells were cultivated on a 12-well plate (1 ^*∗*^ 10^5^ cells/well). After the cells converged to 75%, overexpression of LncRNA ABHD11-AS1 lentiviral vector (ABHD11-AS1-sh), silencing LncRNA ABHD11-AS1 lentiviral vector (ABHD11-AS1-si), LncRNA ABHD11-AS1 empty vector (ABHD11-AS1-NC) and miR-1254 overexpression sequence (miR-1254-mimics), miR-1254 inhibition sequence (miR-1254-inhibition), and miR-1254 negative control (miR-1254-NC) were transfected into cervical carcinoma cells according to Tubfect and LipofectamineTM2000 transfection reagent and were placed at 37°C with 5CO_2_ for continuous culture for 48 h. qRT-PCR was applied to verify the transfection success rate.

### 3.4. qRT-PCR Detection of LncRNA ABHD11-AS1 and miR-1254 Expression

Total RNA was obtained from serum using the RNAiso Plus kit, and tissue and cell samples were digested with pancreatin before extraction. According to the instructions kit, 1 *μ*g of total RNA was reverse transcribed into cDNA. cDNA was amplified according to SYBR Premix Ex Taq™II. Three multiple wells were set up for each reaction. The total reaction system was 20 *μ*L, including 10 *μ*L TBE ×  Taq II (Tli RNase H Plus, 2×), 0.8 *μ*L for forward and reverse primers, 2 *μ*L DNA template, and 6 *μ*L sterile water. PCR reaction conditions: 95°C for 30 s, 95°C for 5 s, 60°C for 30 s, and 50°C for 30 s. GAPDH was applied as the internal reference gene for LncRNA ABHD11-AS1 and U6 for miR-1254. The target gene was calculated by 2^−ΔΔCt^.  Table 1 provides the primer sequence.

### 3.5. MTT Assay Detection of Cell Activity

Cells were cultivated in 96-well plates (1 × 10^5^ cells/well). MTT working solution (50 *μ*L) was put into each well. The cells were cultivated for 72 h in a cell incubator. The supernatant was discarded, and then, 150 *μ*L DMSO was put into each well. The cells were placed on a horizontal shaker and shaken at low speed for 10 min. The absorbance (OD) at 570 nm of each well was read on an enzyme-labeled instrument at 0 h, 24 h, 48 h, and 72 h, respectively, and the cell growth curve was visualized.

### 3.6. Transwell Test Detection of Cell Invasion Ability

Matrix gum was put into the upper chamber of transwell, and complete culture medium was put into the lower chamber. Cells were then put into the upper chamber (3 × 10^4^ cells/well). Cells that did not invade the bottom chamber were washed after 48 hours of culture, and the cells were dyed with 0.2% crystal violet. The number of cells invading the bottom chamber in each field was counted.

### 3.7. Cell Scratch Test Detection for Cell Invasion Ability

After digesting cells with pancreatin, the cells were cultivated into a 6-well plate (1 × 10^6^ cells/well) and cultured until 90% confluent. Scratches were made from top to bottom using a 200 *μ*L pipette tip, followed by incubation for 24 h. The percentage of moving distance of cell front edge was measured by the inverted microscope.

### 3.8. Flow Cytometry Detection for Apoptosis Rate

Trypsin was added to transfected cells for digestion, followed by PBS washing for 2 times, and 100 *μ*L of binding buffer was added to make suspension (1 ^*∗*^ 10^6^ cells/mL). AnnexinV-FITC and PI were put in turn, incubation was conducted in dark for 5 min, and cell apoptosis rate was detected by flow cytometry.

### 3.9. Double Fluorescein Reporters Analysis of the Relationship between LncRNA ABHD11-AS1 and miR-1254

First, the binding sites of LncRNA ABHD11-AS1 and miR-1254 were analyzed by online website ENCORI (https://starbase.sysu.edu.cn/). Subsequently, miR-1254-mimics, miR-1254-inhibition, and miR-1254-NC were transfected into cervical carcinoma cells, and wild-type LncRNA ABHD11-AS1 (ABHD11-AS1-WT) and mutant LncRNA ABHD11-AS1 (ABHD11-AS1MUT) were cloned into pMIR-REPORT luciferase vectors. Cervical carcinoma cells were cultivated into 6-well plates. ABHD11-AS1-WT and ABHD11-AS1MUT sequences were transfected into the cells using Lipofectamine^TM^ 2000. The luciferase activity was tested by the luciferase report detector.

### 3.10. Immunocoprecipitation Experiment Verified the Correlation of LncRNA ABHD11-AS1 with miR-1254

Cervical carcinoma cells were lysed according to the kit instructions and incubated with protein A magnetic beads. After 6 h, the beads were rinsed with washing buffer and then cultivated with 0.1% SDS and 0.5 mg/mL protease K at 55°C for 30 min. The immunoprecipitated RNA was detected by qRT-PCR to prove the existence of LncRNA ABHD11-AS1 and miR-1254.

## 4. Statistical Methods

This experiment was repeated three times. The results were averaged and represented by mean ± SD. SPSS 22.0 was applied for data analysis. The chi-square test was applied for comparison of counting data. The independent sample *t*-test was applied for comparison of measurement data, and the paired *t*-test was applied for comparison before and after treatment. One-way ANOVA and LSD backtesting were applied for comparison among multiple groups. Multiple time points comparison was conducted by repeated measurement analysis of variance and Bonferroni backtesting. Pearson correlation coefficient was applied for correlation analysis. ROC curve was applied to test the predicted value. The survival was tested by Kaplan–Meier method, and the survival was compared by the log-rank test. *P* < 0.05 means a statistically significant difference, while *P* < 0.001 means a significant difference.

## 5. Result

### 5.1. LncRNA ABHD11-AS1 Was Enhanced in Cervical Carcinoma, while miR-1254 Was Reduced

First of all, we detected LncRNA ABHD11-AS1 and miR-1254 in serum of cervical carcinoma patients and healthy people and found that LncRNA ABHD11-AS1 in serum of cervical carcinoma patients was higher than that of healthy people (*P* < 0.05, Figure 1(a)), while miR-1254 was lower than that of healthy people (*P* < 0.05, Figure 1(b)). Subsequently, we detected LncRNA ABHD11-AS1 and miR-1254 in carcinoma tissues and adjacent tissues of cervical carcinoma patients and also found that LncRNA ABHD11-AS1 in carcinoma tissues was higher than adjacent tissues (*P* < 0.05, Figure 1(c)), while miR-1254 was lower than adjacent tissues (*P* < 0.05, Figure 1(d)). Through Pearson correlation coefficient analysis, we found that LncRNA ABHD11-AS1 and miR-1254 expression levels in serum and carcinoma tissues of cervical carcinoma patients were negatively correlated (*P* < 0.05, Figures 1(e) and 1(f)).

### 5.2. High Expression of LncRNA ABHD11-AS1 and Low Expression of miR-1254 Indicated Poor Prognosis of Cervical Carcinoma Patients

After treatment, LncRNA ABHD11-AS1 in serum of cervical carcinoma patients was lower than that before intervention (*P* < 0.05, Figure 2(a)), while miR-1254 was higher than that before intervention (*P* < 0.05, Figure 2(b)). Through 3-year follow-up of prognosis, we successfully followed up 69 patients. Among them, 9 patients died, with a total mortality rate of 13.03% in 3 years. Comparing LncRNA ABHD11-AS1 and miR-1254 after treatment between the dead patients and the survival patients, it was found that LncRNA ABHD11-AS1 in the dead patients was evidently higher than that in the survival patients (*P* < 0.001, Figure 2(c)), while miR-1254 was evidently lower than that in the survival patients (*P* < 0.001, Figure 2(d)). ROC curve revealed that when LncRNA ABHD11-AS1 was more than 6.275 after treatment, the sensitivity and specificity for predicting prognosis death were 88.89% and 90.00% (*P* < 0.001, Figure 2(e)). However, when miR-1254 was less than 3.095 after treatment, the sensitivity and specificity for predicting prognosis death were 88.89% and 83.33%, respectively (*P* < 0.001, Figure 2(f)). Subsequently, we divided the patients into group A (LncRNA ABHD11-AS1 ≥6.275), group B (LncRNA ABHD 11-AS1 <6.275), group C (miR-1254 ≥3.095), and group D (miR-1254 <3.095) according to the expression levels of LncRNA ABHD 11-AS1 and miR-1254 after treatment, and the cutoff value in the above analysis was applied as a boundary. Comparing the survival curve of prognosis among groups, we found that the death rate of prognosis in group A was lower than that in group B (*P* < 0.05, Figure 2(g)), while the death rate of prognosis in group C was higher than that in group D (*P* < 0.05, Figure 2(h)).

### 5.3. Silencing LncRNA ABHD11-AS1 Could Inhibit the Activity of Cervical Carcinoma Cells

First, we detected LncRNA ABHD11-AS1 in HeLa, CaSki, and HcerEpic and found that LncRNA ABHD11-AS1 in HeLa and CaSki was evidently higher than HcerEpic (*P* < 0.001, Figure 3(a)). Subsequently, qRT-PCR was applied to verify the success rate of cell transfection and found that LncRNA ABHD11-AS1 was the highest in the ABHD11-AS1-sh group, followed by the ABHD11-AS1-NC group, and the ABHD11-AS1-si group was the lowest (*P* < 0.001, Figure 3(b)), confirming the success of transfection. The biological behavior test showed that the proliferation, invasion, and migration ability of the ABHD11-AS1-sh group were higher than that of the ABHD11-AS1-si group and ABHD11-AS1-NC group. The proliferation, invasion, and migration ability of the ABHD11-AS1-si group were lower than that of the ABHD11-AS1-NC group (*P* < 0.05, Figures 3(c)–3(f)). The apoptosis rate of the ABHD11-AS1-sh group was lower than that of the other two groups. The apoptosis rate of the ABHD11-AS1-si group was higher than that of the ABHD11-AS1-NC group (*P* < 0.05, Figure 3(g)).

### 5.4. Inhibition of miR-1254 Could Accelerate the Activity of Cervical Carcinoma Cells

After detection, we concluded that miR-1254 in HeLa and CaSki was evidently higher than HcerEpic (*P* < 0.001, Figure 4(a)). qRT-PCR verified the success rate of cell transfection. It was found that miR-1254 was the highest in the miR-1254-mimics group, followed by the miR-1254-NC group, and the miR-1254-inhibition group was the lowest (*P* < 0.001, Figure 4(b)), confirming the success of transfection. Biological behavior examination showed that cell proliferation, invasion, and migration capabilities of the miR-1254-mimics group were lower than those of the miR-1254-inhibition group and miR-1254-NC group, and proliferation, invasion, and migration capabilities of the miR-1254-inhibition group were higher than those of the miR-1254-NC group (*P* < 0.05, Figures 4(c)–4(f)). The apoptosis rate of the miR-1254-mimics group was higher than that of the other two groups. The apoptosis rate of the miR-1254-inhibition group was lower than that of the miR-1254-NC group (*P* < 0.05, Figure 4(g)).

### 5.5. Verification of Targeted Relationship between LncRNA ABHD11-AS1 and miR-1254

LncRNA ABHD11-AS1 and miR-1254 had binding sites through ENCORI (Figure 5(a)). The double fluorescein reporter enzyme experiment found that the fluorescence activity of ABHD11-AS1-WT was hindered by transfected miR-1254-mimics, while the fluorescence activity of ABHD11-AS1-MUT was enhanced by transfected miR-1254-inhibition (*P* < 0.05, Figure 5(b)). However, ABHD11-AS1 and miR-1254 levels precipitated by Ago2 antibody were evidently higher than IgG (*P* < 0.05, Figure 5(c)). Subsequently, we tested miR-1254 in cervical carcinoma cells transfected with ABHD11-AS1-sh, ABHD11-AS1-si, and ABHD11-AS1-NC and found that miR-1254 in the ABHD11-AS1-sh group was lower than that in the ABHD11-AS1-si group and ABHD11-AS1-NC group, and the ABHD11-AS1-si group was higher than the ABHD11-AS1-NC group (*P* < 0.05, Figure 5(d)).

## 6. Discussion

The regulation of LncRNA on the activation process of tumor cells has become a hot topic in clinical research [15, 16]. Its clinical significance mainly lies in the fact that the early screening of tumor diseases still relies mainly on the traditional carcinoma markers CEA and CA199, which cannot accurately respond to complex tumor types, and more and more research studies also show that they can cause abnormalities of carcinoma markers [17]. Therefore, finding specific blood markers is the key to improving the early diagnosis rate of tumors. In addition, the traditional tumor treatment method is mainly surgery or combined with radiotherapy and chemotherapy, which has a good effect on early tumors, but the late patients are still not optimistic [18]. Targeted therapy from the molecular point of view is believed to be better than traditional therapy at home and abroad [19]. Recently, we found that LncRNA ABHD11-AS1 was involved in the occurrence and progression of endometrial carcinoma and also has a regulatory effect on the biological behavior of endometrial carcinoma cells. The study of LncRNA may be the breakthrough for targeted tumor therapy.

First of all, we tested LncRNA ABHD11-AS1 and miR-1254 in the serum of cervical carcinoma patients and healthy people and found that LncRNA ABHD11-AS1 was enhanced, while miR-1254 was reduced. The abnormal LncRNA ABHD11-AS1 and miR-1254 could confirm that they have participated in the development of cervical carcinoma. Subsequently, in order to verify our experimental results, we also detected LncRNA ABHD11-AS1 and miR-1254 in cervical carcinoma tissues and adjacent tissues, and the result was consistent with the above examinations. In addition, we also found abnormal LncRNA ABHD11-AS1 and miR-1254 in other studies, which was consistent with the experimental results [20, 21], indicating that the roles of the two in many diseases can be consistent, and the accuracy of our detection results was confirmed. Subsequently, through correlation analysis, we found that both were negatively correlated in serum and carcinoma tissues of cervical carcinoma patients, which also preliminarily revealed the relationship between the two, indicating that the increase of LncRNA ABHD11-AS1 may cause the decrease of miR-1254, but the specific mechanism is still unclear. We further followed up the prognosis of cervical carcinoma patients in this study for three years, predicted the prognosis and death of LncRNA ABHD11-AS1 and miR-1254 through LncRNA ABHD11-AS1 and miR-1254 after treatment, and found that the effect was extremely excellent, which also showed that the two had certain potential as clinical markers of cervical carcinoma. By observing the survival curve of prognosis, we found that high LncRNA ABHD11-AS1 and low miR-1254 can predict an increase in the prognosis and death of patients, which further indicated that we can effectively evaluate the prognosis of patients by monitoring the changes of LncRNA ABHD11-AS1 and miR-1254 in the future, and carry out effective interventions in a timely and early manner.

In order to understand the exact mechanism of the two in cervical carcinoma, we observed LncRNA ABHD11-AS1 and miR-1254 in cervical carcinoma cells and found that LncRNA ABHD11-AS1 was upregulated and miR-1254 was reduced, confirming the accuracy of our above experiments. Subsequently, we observed the biological behavior changes of cervical carcinoma cells by interfering LncRNA ABHD11-AS1 and miR-1254 and found that silencing LncRNA ABHD11-AS1 could inhibit the activity of cervical carcinoma cells, while inhibiting miR-1254 was the opposite. We can conclude that both LncRNA ABHD11-AS1 with high expression and miR-1254 with low expression play the role of oncogene in cervical carcinoma. Our experimental results also revealed that targeted intervention of LncRNA ABHD11-AS1 or miR-1254 may become one of the effective treatment methods for cervical carcinoma in the future. Of course, more experiments are needed to confirm this. Looking up previous studies, we found that the biological effects of LncRNA ABHD11-AS1 and miR-1254 are the same in pancreatic carcinoma, gastric carcinoma, lung carcinoma, and other diseases [22–24], confirming our experimental results. So far, we have confirmed that LncRNA ABHD11-AS1 and miR-1254 participated in the development and specific role of cervical carcinoma, but the correlation of the two is still not completely clear. In the above, we speculated that LncRNA ABHD11-AS1 may affect the activity of cervical carcinoma cells, which may be related to miR-1254. Therefore, we tested the relationship between the two by double fluorescein reporter enzyme and immunocoprecipitation experiment. The results revealed that LncRNA ABHD11-AS1 and miR-1254 had a targeted regulation relationship, and miR-1254 was increased by silencing LncRNA ABHD11-AS1, while miR-1254 was decreased by overexpressing LncRNA ABHD11-AS1. Therefore, we concluded that LncRNA ABHD11-AS1 accelerated the proliferation, invasion, and migration of cervical carcinoma cells through targeted regulation of miR-1254.

Of course, our research also has many deficiencies and needs further improvement. For example, we have not included patients with cervical benign lesions in this study, and we do not know the specific changes of LncRNA ABHD11-AS1 and miR-1254 in the progression of cervical carcinoma. However, due to the lack of in vitro experimental support, we still need further research on the related signal pathway of LncRNA ABHD11-AS1-targeted regulation of miR-1254. In the future, we will perform more detailed and in-depth tests on the relationship of LncRNA ABHD11-AS1 with cervical carcinoma to improve our experiment.

## Figures and Tables

**Figure 1:** Expression of LncRNA ABHD11-AS1 and miR-1254 in cervical carcinoma. ^*∗*^*P* < 0.05. (a) Comparison of the expression level of LncRNA ABHD11-AS1 in serum of cervical carcinoma patients and healthy people. (b) Comparison of miR-1254 expression level in serum of cervical carcinoma patients and healthy people. (c) Comparison of expression levels of LncRNA ABHD11-AS1 in carcinoma tissues and adjacent tissues of cervical carcinoma patients. (d) Comparison of miR-1254 expression levels in carcinoma tissues and adjacent tissues of cervical carcinoma patients. (e) Correlation analysis of LncRNA ABHD11-AS1 and miR-1254 in serum of cervical carcinoma patients. *r* = −0.517; *P* < 0.001. (f) Correlation analysis of LncRNA ABHD11-AS1 and miR-1254 in carcinoma tissues of cervical carcinoma patients. *r* = −0.691; *P* < 0.001.

**Figure 2:** Clinical significance of LncRNA ABHD11-AS1 and miR-1254 in cervical carcinoma. ^*∗*^*P* < 0.05. ^*∗∗∗*^*P* < 0.001. (a) Comparison of expression levels of LncRNA ABHD11-AS1 in serum of cervical carcinoma patients before and after treatment. (b) Comparison of miR-1254 expression level in serum of cervical carcinoma patients before and after treatment. (c) Comparison of expression levels of LncRNA ABHD11-AS1 between patients with prognosis death and patients with survival. (d) Comparison of miR-1254 expression level between patients with prognosis death and patients with survival. (e) Predictive value of LncRNA ABHD11-AS1 for prognosis and death of cervical carcinoma patients. AUC: 0.904; 95% CI: 0.801–1.0; cutoff: 6.275; sensitivity: 88.89%; specificity: 90.00%; *P* < 0.001. (f) Predictive value of miR-1254 for prognosis and death of cervical carcinoma patients. AUC: 0.907; 95% CI: 0.800–1.015; cutoff: 3.095; sensitivity: 88.89%; specificity: 83.33%; *P* < 0.001. (g) Three-year survival curve of patients in group A and group B. (h) Three-year survival curve of patients in group C and group D.

**Figure 3:** Effect of LncRNA ABHD11-AS1 on cervical carcinoma cells. ^*∗*^*P* < 0.05. ^*∗∗∗*^*P* < 0.001. ^#^Compared with the ABHD11-AS1-sh group, *P* < 0.05. ^&^Compared with the ABHD11-AS1-si group, *P* < 0.05. (a) Comparison of expression levels of LncRNA ABHD11-AS1 in HeLa, CaSki, and HcerEpic. (b) qRT-PCR verified the success rate of cell transfection. (c) HeLa cell proliferation curve. (d) CaSki cell proliferation curve. (e) Invasion of HeLa and CaSki cells. (f) HeLa and CaSki cell migration. (g) Apoptosis rate of HeLa and CaSki cells.

**Figure 4:** Effect of miR-1254 on cervical carcinoma cells. ^*∗*^*P* < 0.05; ^*∗∗∗*^*P* < 0.001. ^#^Compared with the miR-1254-mimics group, *P* < 0.05. ^&^Compared with the miR-1254-inhibition group, *P* < 0.05. (a) Comparison of miR-1254 expression levels in HeLa, CaSki, and HcerEpic. (b) qRT-PCR verified the success rate of cell transfection. (c) HeLa cell proliferation curve. (d) CaSki cell proliferation curve. (e) Invasion of HeLa and CaSki cells. (f) HeLa and CaSki cell migration. (g) Apoptosis rate of HeLa and CaSki cells.

**Figure 5:** Verification of targeted relationship between LncRNA ABHD11-AS1 and miR-1254. ^*∗*^*P* < 0.05. ^#^Compared with the ABHD11-AS1-sh group, *P* < 0.05. ^&^Compared with the ABHD11-AS1-si group, *P* < 0.05. (a) ENCORI analysis of the binding sites of LncRNA ABHD11-AS1 and miR-1254. (b) Detection of fluorescence activity of bifluorescein reporter enzyme. (c) Immune coprecipitation test results. (d) Expression level of miR-1254 in cervical carcinoma cells transfected with ABHD11-AS1-sh, ABHD11-AS1-si, and ABHD11-AS1-NC.

**Table 1:** Primer sequence.

Gene		5′-3′
ABHD11-AS1	Forward	ATGAAGCCATTGCCAAGAAG
	Reverse	GCCTCTCTCTGCAGCTGATT

GAPDH	Forward	GCACCGTCAAGGCTGAGAAC
	Reverse	TGGTGAAGACGCCAGTGGA

miR-1254	Forward	AGCCUGGAAGCUGGAGCCUGCAGU
	Reverse	AGCCUGGAAGCUGGAGCCUGCAGU

U6	Forward	TGGAATCCTGTGGCATCCATGAAAC
	Reverse	TAAAACGCAGCTCAGTAACAGTCCG

## Data Availability

The datasets used and/or analyzed during the current study are available from the corresponding author upon request.
